# Myocardial Remodeling in Diabetic Cardiomyopathy Associated with Cardiac Mast Cell Activation

This article has been retracted.

**DOI:** 10.1371/journal.pone.0060827

**Published:** 2013-03-29

**Authors:** Zhi Gang Huang, Qun Jin, Min Fan, Xiao Liang Cong, Shu Fang Han, Hai Gao, Yi Shan

**Affiliations:** 1 Department of Cardiology, Chang Zheng Hospital, Second Military Medical University, Shanghai, China; 2 Department of Cardiology, The General Hospital of Jinan Military Region, Jinan, China; 3 The Third People's Hospital of Haiyang, Haiyang, Shandong, China; 4 Department of Emergency Medicine, Chang Zheng Hospital, Second Military Medical University, Shanghai, China; Bristol Heart Institute, University of Bristol, United Kingdom

## Abstract

Diabetic cardiomyopathy is a specific disease process distinct from coronary artery disease and hypertension. The disease features cardiac remodeling stimulated by hyperglycemia of the left ventricle wall and disrupts contractile functions. Cardiac mast cells may be activated by metabolic byproducts resulted from hyperglycermia and then participate in the remodeling process by releasing a multitude of cytokines and bioactive enzymes. Nedocromil, a pharmacologic stabilizer of mast cells, has been shown to normalize cytokine levels and attenuate cardiac remodeling. In this study, we describe the activation of cardiac mast cells by inducing diabetes in normal mice using streptozotocin (STZ). Next, we treated the diabetic mice with nedocromil for 12 weeks and then examined their hearts for signs of cardiac remodeling and quantified contractile function. We observed significantly impaired heart function in diabetic mice, as well as increased cardiac mast cell density and elevated mast cell secretions that correlated with gene expression and aberrant cytokine levels associated with cardiac remodeling. Nedocromil treatment halted contractile dysfunction in diabetic mice and reduced cardiac mast cell density, which correlated with reduced bioactive enzyme secretions, reduced expression of extracellular matrix remodeling factors and collagen synthesis, and normalized cytokine levels. However, the results showed nedocromil treatments did not return diabetic mice to a normal state. We concluded that manipulation of cardiac mast cell function is sufficient to attenuate cardiomyopathy stimulated by diabetes, but other cellular pathways also contribute to the disease process.

## Introduction

Diabetic cardiomyopathy is defined as a primary disease process distinct from coronary artery disease and hypertension [1]–[3]. Hyperglycemia contributes to this condition as it induces metabolic disturbances that cause oxidative damage and deregulated cytokine signaling that result in cellular injury, impairment of cell-cell coupling, and apoptosis of myocardial cells. These events, in turn, activate collagen deposition and remodeling of the extracellular matrix [4]. The cumulative result is the stiffening of cardiac tissues that impair normal contractile functions. Therefore, structural abnormalities in the left ventricle (LV), such as interstitial and perivascular fibrosis, are common hallmarks attributed to diabetic cardiomyopathy [4].

Mast cells are recognized as active participants in allergic and anaphylactic reactions [5], [6]. Recent studies showed that mast cells also mediate a wide range of non-allergic reactions including autoimmunity [7], inflammation [8], and infection [9]. Mast cells are tissue-specific and respond to different stimulants in different tissues [10]. The cells function by producing secretory granules that release an assortment of bioactive molecules including cytokines, chemokines, and proteases, such as chymase and tryptase, into the surrounding tissues. In the context of diabetic cardiomyopathy, metabolic byproducts associated with diabetes, such as ROS and oxidized lipoproteins, may trigger mast cell activation [11], but the exact mechanism is unclear because mast cells are sensitive to many environmental stressors and those specific to diabetes have not been identified. However, there are evidence that mast cell activation may contribute, in part, to alterations in cardiac tissue [11]–[13].

There is indirect evidence that cardiac mast cell activation may contribute to cardiac remodeling. Mast cell degranulation has been observed in the human heart [14]. Increased mast cell density has been implicated in human cardiomyopathy [15], and LV fibrosis in hypertensive rat hearts [16]. The biomolecules released by cardiac mast cells may contribute to cardiovascular disease [11], [16]. In particular, chymase has been shown to promote cardiac remodeling by increasing angiotensin II (Ang II) independently from the renin-angiotensin system (RAS) and by altering collagen metabolism [17]–[19]. Furthermore, mast cell density has been associated with MMP activation [20] as chymase was shown to cleave pro-MMP-9 and pro-MMP-2 [21], which may contribute to collagen degradation and remodeling of the cardiac extracellular matrix. Pharmacological inhibition of degranulation using nedocromil (Ned) had not only reduced cardiac remodeling, but also normalized the expression of cytokines such as interferon-γ and tumor necrosis factor-α (TNF-α), as well as anti-inflammatory cytokine interleukin (IL)-4 and IL-10 [16], [22]–[24]. Furthermore, mast cell-deficient rats were protected against adverse cardiac remodeling and showed lower matrix metalloproteinase (MMP) activity, reduced TNF-α activation, and fewer collagen deposits [25].

Based on these previous studies, we propose to use an experimental diabetic cardiomyopathy model to observe if hyperglycemia is associated with cardiac mast cell activation and if mast cell activation correlated with collagen deposition and cardiac remodeling in the heart. We modulate cardiac mast cell activity by administering the mast cell-stabilizing agent nedocromil (Ned) to diabetic mice and then monitor cardiac function, cardiac mast cell activity, expression levels of proteins associated with cardiac remodeling, and the extent of collagen deposition as indirect measurements of the contribution of cardiac mast cell degranulation in diabetic cardiomyopathy.

## Materials and Methods

### Ethic statement

The study protocol was approved by the medical ethics committee of Shanghai Changzheng Hospital, conforms to the Principles of Laboratory Animal Care (National Society for Medical Research), and was conducted according to National Institutes of Health guidelines.

### Animals and treatments

We used previously described methods to induce diabetes in our mouse model [16], [26]. Briefly, 8–12 weeks old C57/BL6 male mice between 23–25 g received intraperitoneal (i.p.) injections of 50 mg/kg streptozotocin (STZ, Sigma, St. Louis, MO), dissolved in 100 mM citrate buffer pH 4.5, for five consecutive days. At 72 h after the final STZ injection, whole blood samples were obtained from the mice using mandibular puncture blood sampling. Blood glucose levels were measured with an Ascensia Counter Glucometer (Bayer health care, NY). Hyperglycemic mice with blood glucose above 15 mmol/L were considered diabetic and were used for our experiments.

Diabetic mice (13-week-old) were randomly divided into three groups: 1) untreated group; 2) nedocromil group, with nedocromil released at the rate of 30 mg/kg per day from a subcutaneous (s.c.) pellet implantation [26]; and vehicle group, with an inactive pellet implanted. Normal mice (non-diabetic) and normal mice that received nedocromil (30 mg/kg per day) were also included in this study for comparison. All sample groups included 15 mice (n = 15).

### Cardiac function assay

To assess cardiac function, mouse hearts were isolated and perfused using the Langendorff system [27] according to published methods [26], [28], [29]. The mice were injected (i.p.) with heparin (10,000 U/kg, Sigma) before the operation. Twenty minutes after the injection, the mice were killed using cervical dislocation. The chest was opened to isolate the heart, which was preserved in ice-cold saline. The perfusion tube was inserted into the aortic root and the heart was perfused with Krebs solution. The solution was maintained at 37°C in a thermostatic water bath with a gas mixture composed of 95% O_2_ and 5% CO_2_ continuously bubbled into the solution. The physiological pressure transducer was sutured to the apical area with 4-0 thread.

Cardiac function indicators were recorded using Powerlab multi-channel physiological recorder. The recorded indicators include maximal contractile rate (+dF/dt), maximal relaxation rate (-dF/dt), heart rate (bpm), and heart work (g.bpm). Heart work was calculated by multiplying the force (g) by the heart rate and normalized to heart weight. After the recording, the left ventricle was placed on ice and then cut transversely into three equal slices perpendicular to the long axis. The slices were either processed immediately for molecular characterization or flash-frozen in liquid nitrogen and stored at -80°C for future analysis.

### Histological characterization

Histological analyses were performed as previously described [30]. Briefly, a slice of the left ventricle was fixed in neutral formaldehyde, embedded in paraffin, and sectioned onto glass slides. The sections were prepared and stained with modified Masson's trichrome to detect myocardial fibers and interstitial fibrosis and estimate collagen deposition. Collagen around blood vessels was not included in the analyses. The collagen volume fraction (CVF) was estimated from five random visual fields of the myocardial interstitium using NIH ImageJ imaging software (version 1.60) and was calculated as the ratio of collagen area/total area. The data shown represent the averaged CVF from five fields.

Immunohistochemical analysis was performed to determine the number of mast cells and mast cell activation based on chymase expression [16], [17]. Briefly, formalin-fixed, paraffin-embedded, 3-μm mouse heart sections were deparaffined in xylol and rehydrated in a graded ethanol series. Antigen retrieval was performed by microwave heating for 20 min in 1 mM EDTA buffer (pH 8.0). The sections were incubated in nonimmune serum for 30 min and then incubated overnight at 4°C in chymase primary monoclonal antibody (dilution 1∶100; Abcam, Cambridge, UK). After washing in TBST, the immunolabeled sections were incubated with HRP-conjugated secondary antibody (dilution 1∶200; Abcam, Cambridge, UK) for 20 min at room temperature, then visualized with 3,3′-diaminobenzidin and counterstained with hematoxylin. The areas of positive and negative staining were calculated using Image-Pro Plus 5.1 software (Media Cybernetics, Silver Spring, MD, USA).

### RT-PCR

Real time-polymerase chain reaction (RT-PCR) was used to measure mRNA expression levels of type I and III collagen, and to confirm chymase mRNA expression. Total cellular RNA was extracted using Trizol (Invitrogen, Carlsbad, CA) according to the manufacturer's instructions. RNA (0.2 µg) was reverse-transcribed using High-Capacity cDNA synthesis kit (Applied Biosystems, California, USA). RT-PCR was performed using the QuantiFast Sybr Green PCR kit (Qiagen, USA). The samples were amplified using Light Cycler 480 real-time PCR machine (Roche Diagnostics, USA). GAPDH expression was used for normalization. mRNA levels were expressed as fold-change relative to untreated normal or untreated diabetic mice. Primers specific for the target genes, the primer's annealing temperature and amplicon length are listed in Table 1.

**Table 1:** Primer sequences, annealing temperatures, and amplicon lengths for RT-PCR.

Target gene	Upstream sequence	Downstream sequence	Length (bp)	Temp. (^o^C)
Type I collagen	5′-TGCCGTGACCTCAAGATGTG-3′	5′-CACAAGCGTGCTGTAGGTGA-3′	462	60
Type III collagen	5′-AGATCATGTCTTCACTCAAGTC-3′	5′-TTTACATTGCCATTGGCCTAG-3′	480	64
Chymase	5′-GAGGCCTGTAAAATCTATAGAC-3′	5′-TGTGTATCTTTGAGAGCCTCAA-3′	351	58
GAPDH	5′-ACGGCAAATTCAACGGCACAGTCA-3′	5′-TGGGGGCATCGGCAGAAGG-3′	231	61

### Western blot

Western blots were used to detect the protein expression levels of type I and III collagen, MMP-2, MMP-9, tryptase, histamine, and chymase in cardiac tissues. Protein extraction was performed using a protein extraction kit (Pierce, Rockford, IL, USA) and the concentration was determined using a protein assay kit (Pierce, Rockford, IL, USA). The extracts were resolved on SDS-PAGE gels by electrophoresis and transferred onto nitrocellulose membranes (Amersham Bioscience, Piscataway, NJ). The membranes were block with 5% nonfat milk in PBS-T. The primary antibodies used were: rabbit anti-mouse collagen I and collagen III antibodies (dilution 1∶5000); rabbit anti-mouse MMP2 and MMP9 antibodies (dilution 1∶1000); rabbit anti-mouse tryptase (dilution 1∶100), rabbit anti-mouse histamine (1∶1000), and goat anti-mouse chymase antibody (dilution 1∶200). Goat anti-rabbit HRP conjugated IgG (dilution 1∶2000), and donkey anti-Goat HRP conjugated IgG (dilution 1∶5000) were used as secondary antibodies to resolve the signal. All antibodies were purchased from Abcam (Cambridge, UK).

### ELISA

Commercial ELISA kits (R&D System, Minneapolis, MN, USA) were purchased to determine the levels of tumor necrosis factor-α (TNF-α), interferon-γ (IFN-γ), interleukin (IL)-6, IL-10, and angiotensin (Ang) II in cardiac tissue. The assays were performed according to manufacturer's instructions using extracted proteins as described above.

### Statistical analysis

Data are expressed as mean ± standard deviation (SD). ANOVA with Scheffe's-F test was used to determine statistical significance between treatment groups, when appropriate. A p-value of <0.05 was considered significant.

## Results

### STZ treatment induced hyperglycemia and weight loss in normal mice

Hyperglycemia has long been implicated in the development of cardiac diseases including cardiac remodeling [1]–[4]. Therefore, we first induced hyperglycemia in normal mice to observe diabetes development and diabetic cardiomyopathy in a controlled manner. We treated C57/BL6 male mice with STZ for five days as previously described, and then monitored blood glucose levels over the following weeks to confirm hyperglycemia.

As shown in Figure 1A, the mice used in the diabetic sample groups displayed a blood glucose level of >15 mmol/L after the final STZ dose, while that of normal mice remained below 10 mmol/L. The diabetic mice then received a continuous dose of nedocromil or vehicle for the next 12 weeks. The glucose levels of the diabetic mice fluctuated between 17 mmol/L and 22 mmol/L during the subsequent weeks. Nedocromil and vehicle treatments did not significantly affect baseline readings in normal or diabetic mice.

**Figure 1:** The blood glucose level and body weight of normal and STZ-induced diabetic mice were monitored for 12 weeks after nedocromil (Ned) treatment, as described in Methods. (A) The blood glucose levels of the different treatment groups at the indicated time points. (B) The body weights of the different treatment groups at the indicated time points. (n = 15 per group).

Figure 1B showed the average body weight of normal and diabetic mice for all treatment protocols. All diabetic mice displayed very similar body weights after the final STZ treatment. However, the body weights between the normal and diabetic mice began to diverge on week 4 as all diabetic mice began to lose weight, while all normal mice began to gain weight. Figure 1B also showed that nedocromil did not affect the baseline body weight of either the normal or the diabetic group.

### Nedocromil significantly improved cardiac function in diabetic mice

Cardiac function was evaluated based on four parameters: maximal cardiac contractility, maximal cardiac relaxation, heart rate, and heart work. Heart work was calculated by multiplying the contraction force by the heart rate and normalized to the heart weight. Figure 2A showed that heart work is significantly lower for hearts in untreated diabetic animals when compared with normal hearts. This observation is likely the result of the lowered magnitude of contractile forces (Figures 2C, 2D), rather than decreased number of heart beats because the heart rate for all mice did not differ significantly (Figure 2B).

**Figure 2:** Cardiac function of isolated and perfused hearts from normal and STZ-induced diabetic mice after nedocromil (Ned) treatments. Contractile function of the heart was determined using a multi-channel physiological recorder. Changes in heart work (A), heart rate (B), maximal rate of contraction (C), and relaxation (D) are presented. Quantitative data are shown as means ± SD (n = 15 per group). *P<0.05 vs. untreated normal group; ^#^P<0.05 vs. untreated diabetic group.

Nedocromil-treated diabetic mice showed significantly improved heart function compared with controls (Figure 2A). The contractility and relaxation forces showed similar improvements (Figures 2C, 2D). However, the cardiac function of nedocromil-treated diabetic mice remained significantly impaired when compared with normal mice (Figures 2A, 2C, 2D). The data indicated that nedocromil can significantly improve cardiac function in mice with diabetic cardiomyopathy, but the treatment cannot restore normal function.

### Mast cell density and activity increased in the hearts of diabetic mice

Previous studies have shown that cardiac mast cells are activated in injured cardiac tissue to mediate cardiac remodeling [15], [16]. Therefore, we decided to probe the cellular and molecular characteristics of cardiac tissues from diabetic mice to assess mast cell activity.

We performed immunohistochemical studies on cardiac tissues from normal and diabetic mice that underwent nedocromil treatment. We examined mast cell activation by assessing chymase level because the enzyme is overexpressed and released during the degranulation process [17].

The number of chymase-positive cells was significantly higher in the cardiac tissues of diabetic mice than in normal mice. Nedocromil significantly reduced the number of chymase-positive cells in samples from diabetic mice, and had little effect on samples from normal mice (Figure 3A, Figure S1). The calculated mast cell density and chymase mRNA expression level reflected a similar trend (Figure 3B, 3C). Overall, the data confirmed mast cell activation in diabetic mice. Nedocromil-treated diabetic mice showed a significant reduction in mast cell number and chymase expression compared with controls, but remained statistically above those of normal mice (Figure 3B, 3C).

**Figure 3:** Characterization of cardiac mast cell activation in normal or STZ-induced diabetic mice after nedocromil (Ned) treatments. (A) Quantification of chymase-positive mast cells. Chymase-positive cells from immunohistochemically stained cardiac tissues were counted in 100 random fields at 400X magnification. (B) Mast cell density in sample tissues was determined by dividing the number of chymase-positive cells by the total number of cells in the visual fields. (C) mRNA expression levels of chymase in sample tissues were normalized to GAPDH expression and depicted as fold-change relative to the untreated normal group. (D) Representative results of protein expression analysis for chymase, tryptase, and histamine in sample tissues using western blot. GAPDH expression is shown as loading control. Quantitative data are displayed as means ± SD (n = 15 per group). ^*^P<0.05 vs. untreated normal group; ^#^P<0.05 vs. untreated diabetic group.

We further confirmed cardiac mast cell activation by evaluating the protein levels of additional mast cell-associated enzymes, which are also induced upon mast cell activation [11], [16]. The western blot in Figure 3D showed an increase in chymase, tryptase, and histamine that corresponded with diabetes and mast cell activation. The addition of nedocromil induced a modest decrease in the chymase level of diabetic and normal mice compared with vehicle-treated control, but no significant reduction of tryptase or histamine was observed in diabetic or normal mice (Figure 3D). This observation suggests that the modulatory effect of nedocromil is limited and degranulation was not completely blocked.

### Nedocromil treatment decreases factors associated with cardiac remodeling

We have observed nedocromil treatment improved overall cardiac function in diabetic mice (Figure 2). So, we examined the expression profile of factors associated with cardiac remodeling to determine whether the functional improvements correlated with decreased remodeling. We used the expression of type I and type III collagen to monitor collagen deposition. We also measured MMP-2 and MMP-9 protein expression, which were reported to modulate the extracellular matrix by degrading collagen and were associated with cardiac remodeling [26], [31].

Trace amount of collagen deposits were observed in the hearts from normal mice, while those from diabetic mice showed significant areas of collagen deposition (Figures 4A, 4B) that correlated with molecular characterization (Figures 4A, 4B). MMP-2 and MMP-9 were also overexpressed, which suggested a high rate of collagen turnover in diabetic mice that may indicate active cardiac remodeling. Nedocromil treatment significantly reduced collagen deposits and MMP-2 and -9 expression levels in diabetic mice when compared with controls, but they remained greater than in normal mice (Figures 4A, 4B). Nedocromil may have stabilized collagen turnover and halted cardiac remodeling associated with diabetic cardiomyopathy.

**Figure 4:** Collagen deposits in the left ventricle (LV) of normal and STZ-induced diabetic mice after nedocromil (Ned) treatments. (A) Representative images of LV sections stained with Masson's trichrome at 100X magnification. Blue color indicates collagen deposits. (B) Quantification of LV collagen volume fraction (CVF). CVF is represented as the ratio of collagen area/total area. (C) The mRNA expression levels of type I and type III collagen are normalized to GAPDH expression and depicted as fold-change relative to the untreated normal group. (D) Representative results of protein expression analysis for collagen I, collagen III, MMP-2, and MMP-9 in sample tissues using western blot. GAPDH expression is shown as loading control and used for normalization. (E) Quantification of type I and type III collagen, MMP-2, and MMP-9 protein levels normalized to GAPDH. Quantitative data are displayed as means ± SD (n = 15 per group). ^*^P<0.05 vs. untreated normal group; ^#^P<0.05 vs. untreated diabetic group.

### Nedocromil treatment modulated cytokines associated with cardiac remodeling in diabetic mice

Cardiac mast cell activation was reported to modulate cytokines that contribute to cardiac remodeling [16]. Therefore, we evaluated the extent to which mast cell activation modulate various cytokine levels in the heart. We used commercial kits to quantify several pro-inflammatory cytokines—specifically tumor necrosis factor-α (TNF-α), interferon-γ (IFN-γ) and also anti-inflammatory cytokine interleukin (IL)-4 and IL-10, which was reported to block inflammation and attenuate left ventricle remodeling [32]. We also evaluated angiotensin II, which is a cytokine-like factor known to mediate cardiac remodeling and is produced primarily by chymase in the heart, rather than by the RAS [18], [19].

Figures 5A and 5B showed diabetic mice had significantly higher levels of TNF-α and IFN-γ than normal mice. Nedocromil treatment was able to significantly decrease TNF-α and IFN-γ in diabetic mice relative to control. The levels of IL-4 and IL-10 were significantly reduced in diabetic mice compared with normal mice (Figures 5C, 5D). This pattern is consistent with the known anti-inflammatory properties of IL-4 and IL-10 [22]–[24]. Nedocromil treatment reversed this trend and the expression of both cytokines increased in diabetic mice to normalized levels (Figures 5C, 5D). Ang II was induced in diabetic mice, and nedocromil treatment was able to significantly reduce Ang II levels in diabetic mice relative to vehicle-treated control (Figure 5E). The results suggested nedocromil has indirect modulatory effects on cytokine levels by stabilizing mast cell activity.

**Figure 5:** ELISA assay for cytokine expression in cardiac tissues of normal and STZ-induced diabetic mice treated with nedocromil (Ned) or controls. The graphs show the quantitative levels of (A) TNF-α, (B) IFN-γ, (C) IL-4, (D) IL-10, and (E) Angiotensin II (Ang II) of the indicated sample groups. Quantitative data are displayed as means ± SD (n = 15 per group). ^*^P<0.05 vs. untreated normal group; ^#^P<0.05 vs. untreated diabetic group.

## Discussion

Hyperglycemia has long been implicated in cardiac diseases by producing metabolic stress and triggering cardiac remodeling [1]–[4]. Mast cells have been suggested to regulate cardiac fibrosis by Panizo et al. [33], and later studies bolstered the claim by showing cardiac mast cell activity was stimulated in injured cardiac tissue to mediate cardiac remodeling [15], [16]. The cumulative evidence suggests cardiac mast cell activation is correlated with cardiomyopathy, but the role of hyperglycemia in cardiac mast cell activation remains unclear.

We have presented data that showed cardiac mast cell activation and cardiac remodeling occurs following hyperglycemia. The hearts of STZ-induced diabetic mice showed significantly impaired contractile function that resulted from increased collagen deposits and initiation of extracellular matrix degradation. We also examined chymase and tryptase levels in the heart because the enzymes are known mast cell products and have been linked to increased collagen production and to induce remodeling of the extracellular matrix by cleaving pro-forms of MMP-2 and MMP-9 [17], [19], [21], [34], [35]. We confirmed that mast cell numbers and protease production were significantly increased in hyperglycemic mice, which is consistent with a previous study [36]. Taken together, we speculate that mast cell activation and protease secretion may be responsible for cardiac remodeling by increasing collagen turnover, which in turn, destabilizes the cardiac extracellular matrix in diabetic mice. When this phenomenon is combined with the mechanical forces in a beating heart, it may be sufficient to induce cardiac remodeling and disrupt cardiac functions.

Many of these features were reversed upon mast cell stabilization using nedocromil. We showed the drug had protective effects against cardiac dysfunction in diabetic mice by reducing mast cell density and chymase secretion, and confirmed the expression of remodeling factors had decreased using biochemical assays.

We also observed aberrant cytokine levels in diabetic mice, which may contribute to cardiac remodeling. Nedocromil treatment was able to normalize them in diabetic mice. Cardiac mast cell activation has been reported to modulate cytokines that contribute to cardiac remodeling [16], [18], [19], and our results support this idea in the context of hyperglycemic mice.

Tumor necrosis factor-α (TNF-α), interferon-γ (IFN-γ), and angiotensin Ang (II) have long been associated with cardiac remodeling. They were all significantly increased in diabetic mice. TNF-α is known to increase collagen production by stimulating the angiotensin II type 1 receptor [37], while knockout experiments showed TNF-α is required for cardiac remodeling under hypertensive conditions [38]. IFN-γ expression was also increased in our diabetic mice. IFN-γ is a marker not only of mast cell activation, but is also used to identify T-cell activation [39]. This is interesting because it suggests other factors may also modulate IFN-γ expression and extracellular matrix remodeling [40]. In fact, this is likely the case because nedocromil treatment was able to improve cardiac function in our model, but not restore normalcy. Ang II production is primarily mediated by chymase in the heart [18], [19], which further support mast cell activation and chymase secretion in diabetic mouse hearts. Nedocromil treatment reduced the expression levels of both chymase and Ang II, suggesting the drug may reduce Ang II levels indirectly via chymase inhibition.

The role of IL-6 in cardiac remodeling is unclear because its expression has been shown to vary greatly at different stages of cardiac remodeling in hypertensive rats [41], [42]. Its role is further complicated by the modulatory effects exerted by anti-inflammatory cytokine IL-10 [22]–[24], which was significantly decreased in diabetic mice and increased after nedocromil treatment.

Our data also showed nedocromil had no effect on blood glucose levels in diabetic mice, indicating mast cell activation is likely correlated with blood glucose levels and not by possible nonspecific effects from nedocromil. We also confirmed the effects of nedocromil had no significant effects in normal mice. However, the drug did not completely inhibit the degranulation process, as shown by the stable tryptase and histamine levels. We speculate that heightened levels of tryptase and histamine in diabetic mice may contribute to cardiac remodeling by an unknown mechanism, which may explain why nedocromil treatment did not completely abrogate the molecular changes observed in diabetic hearts.

We have shown a correlation between mast cell activation and cardiac remodeling in diabetic mice. We concluded that regulating mast cell activity was sufficient to significantly improve heart function in diabetic mice, and reduce signs of collage deposition and extracellular matrix destablization. Nedocromil treatment alone normalized the levels of several cytokines that are known contributors to cardiac remodeling. Our results propose that the manipulation of cardiac mast cells can attenuate cardiomyopathy by modulating aberrant cytokine levels. However, this mechanism is insufficient to fully restore normal cardiac functions and suggests other cellular pathways may contribute to the disease process. In addition, the molecular mechanisms that link hyperglycemia and cardiac mast cell activation remain unclear and warrant further study.

## Supporting Information

Figure S1 **Immunohistochemical staining for chymase in cardiac tissues (400X magnification).**
(TIF)
